# Futuristic Developments and Applications in Endoluminal Stenting

**DOI:** 10.1155/2022/6774925

**Published:** 2022-01-11

**Authors:** Joel Ferreira-Silva, Renato Medas, Mohit Girotra, Monique Barakat, James H. Tabibian, Eduardo Rodrigues-Pinto

**Affiliations:** ^1^Gastroenterology Department, Centro Hospitalar São João, Porto, Portugal; ^2^Faculty of Medicine of the University of Porto, Porto, Portugal; ^3^Digestive Health Institute, Swedish Medical Center, Seattle, Washington, USA; ^4^Division of Gastroenterology, Stanford University, California, USA; ^5^Division of Gastroenterology, Department of Medicine, Olive View-UCLA Medical Center, Sylmar, CA, USA; ^6^UCLA Vatche and Tamar Manoukian Division of Digestive Diseases, David Geffen School of Medicine at UCLA, Los Angeles, CA, USA

## Abstract

Endoscopic stenting is a well-established option for the treatment of malignant obstruction, temporary management of benign strictures, and sealing transmural defects, as well as drainage of pancreatic fluid collections and biliary obstruction. In recent years, in addition to expansion in indications for endoscopic stenting, considerable strides have been made in stent technology, and several types of devices with advanced designs and materials are continuously being developed. In this review, we discuss the important developments in stent designs and novel indications for endoluminal and transluminal stenting. Our discussion specifically focuses on (i) biodegradable as well as (ii) irradiating and drug-eluting stents for esophageal, gastroduodenal, biliary, and colonic indications, (iii) endoscopic stenting in inflammatory bowel disease, and (iv) lumen-apposing metal stent.

## 1. Introduction

Endoscopic stents are hollow devices designed to prevent constriction or collapse of a tubular portion of gastrointestinal (GI) tract and currently used in management of variety of diseases of the esophagus, stomach, small bowel, colon, and bilio-pancreatic system. Common indications of endoscopic stents include reestablishment or maintenance of luminal patency in cases of malignant obstruction and temporary treatment of benign strictures, as well as sealing transmural defects and diverting luminal contents in leaks, fistulae, or perforations [1]. GI stents were originally designed as rigid, cylinder-like prostheses and, as a result, had poor efficacy and high adverse event rates [1]. However, stent design has been subject to continuous improvement.

In recent years, in addition to expansion in indications for endoscopic stenting, considerable strides have been made in stent technology, and several types of devices with advanced designs and materials are continuously being developed. In this review, we discuss the important developments in stent designs and novel indications for endoluminal and transluminal stenting. Our discussion specifically focuses on (i) biodegradable as well as (ii) irradiating and drug-eluting stents for esophageal, gastroduodenal, biliary, and colonic indications, (iii) endoscopic stenting in inflammatory bowel disease (IBD), and (iv) lumen-apposing metal stent (LAMS).

## 2. Biodegradable Stents

Self-expandable metal and plastic stents (SEMS and SEPS, respectively) are an effective treatment option in the management of both benign and malignant strictures, as well as leaks and fistulae, throughout the GI tract [2, 3]. However, the use of these stents is associated with several common problems, such as stent migration, blockage, and tissue ingrowth, thus requiring repetitive endoscopic procedures. To overcome the shortcomings of SEMS and SEPS, biodegradable stents (BDS) with GI tract applications have been developed. BDS may be particularly useful in benign pathology, as well as clinical situations wherein the stent is needed temporarily, by obviating the need of a follow-up procedure typically required for stent removal. Moreover, BDS may also be associated with lower rates of stent migration and tissue ingrowth, thus offering additional advantages over SEMS. However, the radial force of BDS is weaker than that of SEMS and also requires manual mounting on a delivery system for deployment, making the process complicated compared to SEMS, which are available preassembled and ready-to-use [4]. Other disadvantages of BDS include significant stent shortening and radiolucency, except for added markers, thus making deployment challenging.

Different biomaterials with varied characteristics are used to manufacture BDS, most common being synthetic polymers: polylactide, polydioxanone (PDX), polycaprolactone, and poly-lactide-co-glycolide with self-expandable design [5]. Although no data exists comparing BDS stents manufactured from different biodegradable polymers, as a biodegradable material, PDX may have superior flexibility, degrade more slowly by hydrolysis, and retain its biomechanical properties longer than other polymers [6]. Usually, the radial force of BDS stent is maintained for 6 weeks following deployment, and the stent degrades in 6-24 weeks. Different BDS designs have been developed with applications in esophageal, small bowel, colonic, and pancreatobiliary tract pathology, as discussed below.

### 2.1. Biodegradable Stents in the Esophagus

BDS offer an emerging and promising treatment alternative in patients with benign esophageal strictures. Dilation is currently the standard of care in this context, allowing dysphagia improvement in the majority of patients [7]. However, repeated sessions are frequently required, and some strictures are refractory to dilations [7, 8]. In patients with refractory strictures, stent placement is an alternative treatment, wherein stricture remodelling due to indwelling stent results in improved luminal patency during the remission of the underlying inflammatory process [9]. Partially covered (PC) and fully covered (FC) SEMS have been traditionally used in such situations but present several limitations including stent migration, tissue ingrowth, and/or requirement for additional endoscopic procedures for stent removal [10]. The use of BDS has been suggested to overcome these limitations (Figures 1(a) and 1(b)), but compelling evidence for use of BDS over other stent types is still lacking [11–17]. The rationale behind BDS consists of a constant radial force applied for a specific amount of time (6–8 weeks), with concurrent progressive hydrolysis-mediated self-degradation (8–12 weeks), thus avoiding both the development of tissue overgrowth as well a need for repeat endoscopic procedure for stent removal.

Currently, PDX BDS, loaded manually prior to placement onto a 28Fr delivery system, not compatible with through-the-scope (TTS) placement technique, is the only commercially available BDS for esophageal use. Dhar et al. and Walter et al. compared BDS to endoscopic balloon dilatation (EBD) in two RCTs with 17 patients and 66 patients, respectively [16, 17]. The former study showed that stenting was associated with greater dysphagia scores, need of comedication and adverse events, thus not supporting use of BDS. On the contrary, the latter study showed that the BDS group (*n* = 32) underwent significantly less endoscopic dilations for recurrent stricture compared to the EBD group (*n* = 34) in initial 3 months, while this effect was lost by 6 months. This temporary benefit may reduce healthcare costs and improve the quality of life as a transient palliative intervention. However, in studies comparing different stent designs [15], all types of self-expandable stents appear to offer only modest (30-40%) rates of long-term dysphagia relief. Dysphagia recurrence, poststenting chest pain, and tissue hyperplasia were the most commonly reported adverse events [15]. In a meta-analysis of 18 studies (10 prospective, 8 retrospective studies; 444 patients), the efficacy and safety of expandable stenting (BDS, SEMS, or SEPS) for refractory benign esophageal stricture (RBES) were evaluated [13]. The pooled clinical success was 40.5%, migration rate was 28.6%, and overall complication rate was 20.6%. No statistically significant differences were noticed between the 3 groups in overall clinical success, stent migration, and complication rates. Considering these data, the updated European Society for Gastrointestinal Endoscopy (ESGE) guidelines do not recommend a specific type of stent (FCSEMS, SEPS, or BDS) since none have shown to be superior to any other for this indication [18]. The development of new esophageal BDS with different polymeric mixtures, currently available only for biliopancreatic diseases, could represent an attractive therapeutic option in the future, for the purpose of refractory benign esophageal stricture (RBES) management [19].

The role of BDS in the management of malignant esophageal strictures is not adequately defined, and in such scenarios, BDS is not yet considered a valid alternative to SEMS. Studies have evaluated outcomes of BDS in patients undergoing single dose brachytherapy [20], palliative radiotherapy [21], and neoadjuvant treatment or radical radiotherapy [22], but in each of these studies, despite adequate technical success and short-term dysphagia symptom improvement, unacceptably high rates of adverse events and complications (retrosternal pain, vomiting, epithelial hyperplasia, and stent-related death), stent dysfunction, and need for reintervention were reported [20–22]. To overcome these limitations, BDS using novel materials (elastic and biodegradable mixed polymer of Poly(*ε*-caprolactone) (PCL) and poly(tri-methylene carbonate) (PTMC) as the coated membrane on magnesium alloy stents) are being developed but have not yet been tested in humans [23, 24].

Regarding role of BDS in management of esophageal transmural defects (Figures 1(c) and 1(d)), the data is limited, with only two studies, comprising of 13 and 4 patients, wherein the clinical success ranged from 77.8 to 100%, but a drawback of mucosal reaction (2/4 patients) causing dysphagia requiring endoscopic dilation [25, 26].

### 2.2. Biodegradable Stents in the Small Bowel and Colon

Different studies have evaluated the safety and efficacy of BDS in the treatment of benign strictures in small bowel and colon, as well as for management of anastomotic colorectal strictures, stricturing Crohn's disease (CD), and postsurgical colonic fistulae [27–32]. The most common stent in this context is PDX BDS, initially developed for esophageal use, and as stated previously, it is not compatible with TTS deployment. Additionally the standard delivery system of PDX BDS with an active length of 75 cm precludes proximal colonic stent placement or in patients with considerable colonic angulation/tortuosity due to technical challenges [31].

The largest series of BDS stents in colon and ileocolic anastomotic strictures report a technical success of 90-100% but only a modest stricture resolution of 45-83% [28, 31], with early stent migration being the main reason for clinical failure. Unlike in esophageal strictures, mucosal hyperplastic reaction after BDS placement has not been reported in intestinal strictures. The use of BDS in CD strictures is discussed in greater detail in a different section of this article.

### 2.3. Biodegradable Stents in the Pancreatobiliary Tract

The use of BDS during endoscopic retrograde cholangiopancreatography (ERCP), until recently, was only reported in animal models [33–35]. In 2015, an insertion device enabling TTS deployment (diameter of 3.9 mm) compatible with PDX self-expandable BDS was developed. This technology was successfully tested first in a postoperative cystic duct biliary leak patient [36]. Subsequently, the same group of authors expanded the use of PDX BDS for benign biliary strictures, in addition to cystic duct leaks [37]. While all bile leaks (*n* = 7) healed successfully, the authors reported 83% clinical success in benign stricture (*n* = 6) treatment with median follow-up of 21 months (range 14-25). No early stent migrations or dysfunction were observed, and the stents degraded as expected in 3–6 months. However, mild acute cholangitis was reported in 3/13 (23%) patients within 90 days poststent deployment. Interestingly, similar high rates of mild acute cholangitis were reported with percutaneously placed PDX BDS as well [38]. Siiki et al. evaluated 32 patients prospectively, comparing plastic stents (*n* = 24) and BDS (*n* = 8) in the treatment of postcholecystectomy bile leak [39] and noted no statistical difference in the clinical success rate, rates of readmission, or 30-day adverse event rate (13% in both groups), although total drain output was lower in BDS patients (330 ml vs. 83 ml, *p* = 0.002). All patients with BDS were spared repeated endoscopy for stent removal.

Lindström et al. reported their experience of BDS in 7 patients with Roux-en-Y hepatojejunostomy anatomy, for management of HJ strictures (*n* = 3) or intrahepatic strictures (*n* = 4) [40]. The authors noted stricture resolution in all cases, without any stent or cholangiography-related complication, and one stent migration in 90-day follow-up. More recently, a new helicoidal BDS with pancreatobiliary application has been described [19], with a nonexpandable design and the deployment mechanism similar to plastic stents, available in different sizes and variable rates of biodegradability, depending on the composition of the polymeric mixtures. Main indications of this new stent include prevention of post-ERCP cholangitis and postcholecystectomy bile duct stricture management, and the only adverse event reported was 1 post-ERCP pancreatitis, although premature stent migration occurred in 9.4% of the patients.

## 3. Irradiating and Drug Eluting Gastrointestinal Stents

SEMS have shown significant clinical success in the palliation of GI malignancies and are commonly used in the management of esophageal, gastric, duodenal, pancreatico-biliary, and colorectal obstructive neoplasia. However, these conventional stents can suffer from stent obstruction due to tumor and/or tissue ingrowth and/or overgrowth [41]. To overcome this limitation, there is growing interest in the development of irradiating and drug-eluting stents (DES), which can provide a sustained and localized release of drugs, which minimize tumor/tissue growth to optimize stent efficacy. As such, several stent designs that combine the mechanic characteristics of SEMS with different types of drugs have been developed, for clinical use in patients with esophageal and biliary malignancies [42].

Only a limited number of clinical trials have evaluated the role of irradiating and DES in patients with inoperable esophageal cancer-related dysphagia. In 2017, a meta-analysis (3 RCTs, 3 observational studies; 539 patients) by Chen et al. comparing traditional SEMS versus radioactive SEMS (loaded with iodine-125 seeds) or SEMS with brachytherapy [43] showed that SEMS with brachytherapy had a longer overall survival (2.7 months), as well as improved survival at 1, 3, and 6 months. Both stent types resulted in good immediate dysphagia relief, but radioactive stent performed better at 3 and 6 months of follow-up, without significant differences in complication rates. Moreover, a more recent meta-analysis in 2020 (6 RCTs; 403 patients) compared traditional SEMS with radioactive SEMS (loaded with iodine-125 seeds) [44] and showed no significant difference between the two stent types in either the dysphagia scores or stent restenosis, migration, severe chest pain, and other complications (hemorrhage, fistula formation). However, time to restenosis and overall survival were better in the radioactive stent group [45]. Several retrospective studies have also concurred that radioactive SEMS have a longer stent patency [45, 46] and better survival [45–47] with similar complication rates compared to traditional SEMS, albeit at a higher cost [48].

Following the huge clinical success of drug-eluting vascular/cardiac stents, there has been a significant curiosity in other applications of DES, including treatment of GI cancers [49]. While new DES utilizing various drugs (docetaxel, 5-fluorouracil, paclitaxel, or gemcitabine) combined with different types of stent construction technologies (such as 3D printing) and different varieties of polymer coatings are being developed [41, 48, 50–53], currently, there are no clinical data in humans for use of these DES for palliation of esophageal cancer.

The role of irradiating stents in the treatment of malignant biliary obstruction (MBO) has also been recently evaluated. Zhu et al. performed a randomized trial of 328 patients with unresectable MBO and found a longer patency time of irradiating stents (212 days) when compared to uncovered SEMS (104 days) [54]. Also, irradiating stents were significantly associated with decreased rates of stent restenosis and longer survival time (median 202 days vs. 140 days; *p* = 0.020), but no differences in technical success rate or rates of complications. DES have also been developed for MBO in an attempt to improve long-term stent patency of SEMS due to tumor ingrowth; however, there is a paucity of human data in this regard. Studies on paclitaxel eluting stents [55–57] consistently report no differences in survival or stent patency rates compared to covered metal stents, albeit with possibly higher rates of stent migration [57]. Similarly, a meta-analysis of five prospective studies evaluating efficacy of paclitaxel-eluting stents compared to SEMS [58] found no differences in pooled stent patency (OR 1.03, *p* = 0.9), overall survival (OR 1.16, *p* = 0.6), or adverse events. Another meta-analysis reported similar rates of survival and stent patency, but higher frequency of cholangitis-like symptoms in the DES group [59]. These suboptimal outcomes of DES may be due to the fact that dual chemotherapy (cisplatin and gemcitabine) may be more effective than paclitaxel alone [60]. Other DES using sorafenib and gemcitabine appear promising in vitro and in porcine models, though human studies are necessary to confirm their efficacy and safety [61, 62].

Finally, a few recent studies have evaluated the efficacy of polyglycolic acid sheet combined with covered SEMS for prevention of stricture formation after large esophageal endoscopic submucosal dissection (ESD) [63–65]. The rate of post-ESD esophageal stricture appears to be lower in patients treated with polyglycolic sheet SEMS when compared to patients treated with conventional SEMS or intralesional steroid injection, with similar safety profile, making it a promising alternative in this context.

## 4. Stents in Inflammatory Bowel Disease

Strictures are one of the most frequent complications of CD, occurring in up to a third of patients within 10 years of diagnosis, as a result of underlying disease, surgical anastomosis, or previous stricturoplasty [66]. Strictures in CD are more frequently localized in the small bowel rather than in the colon (64% vs. 5%, respectively). Bowel resection and stricturoplasty are effective for the treatment of primary or secondary (i.e., anastomotic) strictures; however, within 4 years after initial ileocolic resection, over 40% patients have recurrent obstructive symptoms [67], besides the risk of postoperative complications associated with the invasive nature of surgical therapies. This high rate of recurrence suggests that conservative treatment should be preferred in order to avoid repeated surgery.

Currently, the endoscopic treatment of choice of CD strictures is EBD [68]. Several studies have proven safety and efficacy of EBD for primary or anastomotic strictures ≤4–5 cm in length, with success rates of 44-58% [69–71]; however, post EBD relapse requiring reintervention ranges from 46% to 62% [72, 73]. Therefore, patients with a poor immediate response or an absence of long-term efficacy could benefit from alternative endoscopic treatments or surgery. In these patients, endoscopic stents could represent a minimally invasive alternative.

Data regarding safety and efficacy of SEMS in the context of CD strictures is limited and inconclusive. Our literature review has identified 20 publications (mostly case reports/small series) with 71 patients [32, 74–86], wherein majority of patients with colonic or ileocolic anastomotic stricture previously treated with EBD were managed using FC-SEMS or PC-SEMS with a clinical success rate of 36-100%. Patients who achieved clinical success remained symptom free for up to 10-12 months of follow-up, with mean stenting duration being 28 weeks. Major adverse events included stent migration (especially with FC-SEMS and associated with stricture resolution), perforation in 2 patients (both with stent dwell time longer than 100 weeks), and technically difficult stent removal (especially with PC-SEMS). The largest of these series by Loras et al. in patients with ileocolonic anastomotic strictures treated with 20 mm diameter FC-SEMS, maintained for an average of 28 days showed treatment efficacy in 64.7% patients, with 1 adverse event (proximal stent migration) [87].

Das et al. evaluated the efficacy of seven-day stenting in 21 CD patients with terminal ileum or ileocolonic anastomosis stricture and noted symptom improvement in 81% patients, with only 5 reported adverse events (2 stent-related discomfort, 3 asymptomatic stent migrations) and no requirement for stricture-related surgery during follow-up (3-50 months) [88]. Hedenström and Stotzer compared 20 mm diameter SEMS (*n* = 7) and 18 mm balloon dilation (*n* = 5) in patients with symptomatic ileo-cecal stricture and noted significantly higher clinical success (defined as no need for repeated interventions) in the stent group (86%) compared to dilation alone (20%) [89]. However, the study was terminated preterm following the higher incidence of adverse events in the stent group (mainly pain and rectal bleeding in 53% of patients).

While BDS can theoretically avoid the shortcomings of SEMS, mainly stent migration and the need for stent removal, however, the absence of biodegradable TTS colonic stents makes deployment proximal to the sigmoid technically challenging. Data is very limited in this context [31, 85, 87, 90]. Rejchrt et al. reported a series of 11 patients with CD strictures of the terminal ileum or colon, in whom BDS stents were deployed through an overtube, assisted by a stiff guidewire and with fluoroscopy guidance, with high technical success (90.9%), but early stent migration (between 2 days and 8 weeks) in 3/11 patients [32].

## 5. Lumen-Apposing Metal Stents (LAMS)

The LAMS designed for transluminal drainage was first described in 2011 [88]. The unique design of LAMS combined with the properties of a FC stent allows direct apposition of two separate lumens with minimal risk of leakage of enteric contents [88]. Furthermore, the large stent diameter gives the additional advantage of allowing direct endoscope manipulation of the bridged lumen. Several LAMS designs are commercially available. Teoh et al. performed an ex vivo comparison of the lumen-apposing force (LAF) of 3 designs of available LAMS [91]. In this study, LAFs were significantly higher for stents A (Axios) and S (Spaxus) when compared with stent N (Nagi) (*p* < 0.001).

LAMS are now a well-established indication for drainage of pancreatic fluid collections, due to their safety and efficacy profile. Several meta-analyses have evaluated LAMS for the drainage of pancreatic collections [92, 93], with technical and clinical success of 98.9% and 90% for walled-off pancreatic necrosis and 97% and 98% for pancreatic pseudocysts [93], with an adverse event rate of 11%. LAMS have also been compared to plastic stents in this context [92], with better clinical success (pooled RR of 0.37) and better safety profile (pooled RR of 0.39).

### 5.1. Drainage of Abdominopelvic and Mediastinal Collections

Besides management of pancreatic fluid/necrosis collections, creation of a fistula for drainage of an infected cavity can theoretically be performed in any part of the accessible GI tract, as long as the collection is in close proximity with the GI wall. Percutaneous or surgical drainage of abdominal or mediastinal collections have been the standard of care till now; however, percutaneous approach is marred with shortcomings of an external drain, including dislodgement, blockage, leakage, and hence requiring additional procedures [94], while surgical drainage is usually reserved for patients with inaccessible collections or those who fail to improve with percutaneous drainage. EUS-guided drainage of abdominopelvic and mediastinal collections is evolving into a promising alternative; however, data regarding safety and efficacy is still limited.

EUS-guided drainage of mediastinal collections with LAMS (Figure 2) has been described in several case reports [95–98]. Transesophageal drainage was technically successful in all five patients reported in these series, without any major complications. Naso-esophageal tube was placed in 2 patients, and LAMS was left in place for 3-7 days, with esophageal fistula clip closure in all patients after LAMS removal [96–99]. EUS-guided drainage of abdominopelvic collections with LAMS is slightly better reported [99, 100]. The largest case series included 47 patients [100], where fluid collection secondary to pancreatic duct leak after pancreatic resections was the foremost cause, along with other postsurgical collections (liver transplantation, liver resection, cholecystectomy, colorectal resection, gynecologic surgery, and bariatric surgery). Drainage route was transgastric in the majority of patients, with transduodenal and transrectal access utilized in 5 and 8 patients, respectively. Overall technical and clinical success was 93.6% and 89.3%, respectively, with intraprocedural (stent migration) and postprocedural adverse events (1 migration, 1 perforation, 1 infection) in 4.25% and 6.4% of the patients, respectively [100, 101].

Finally, the role of EUS-guided plastic stent drainage of pelvic abscess has also been evaluated. A recent meta-analysis by Dhindsa et al. evaluated 8 studies with 135 patients with pelvic abscesses of different etiologies (mainly postsurgical and diverticulitis), with mean size 63.32 mm, and 83.7% being peri-rectal and remainder peri-colonic in location [101]. Drainage was performed with double-pigtail plastic stents and was reported technically successful in 100%. The calculated pooled rate of clinical success was 92% and 9.4%, adverse events with stent migration (5.5%) being the foremost.

### 5.2. Gastro-Enteric and Entero-Enteric Anastomosis

EUS-guided gastro-enteric (GE) and entero-enteric (EE) anastomosis is an emerging technique in selected cases of gastric outlet obstruction (GOO), afferent loop syndrome (ALS), and patients who failed ERCP due to altered anatomy [102, 103]. The rationale of EUS-guided GE is similar to surgical gastro-jejunostomy (SGJ) and consists in identifying the target jejunal loop, followed by the creation of a gastro-jejunal or jejuno-jejunostomy under ultrasonographic and endoscopic visualization. Bi-flanged LAMS, particularly those with electrocautery-enhanced delivery systems, are the most used devices to create the GE anastomosis, and its availability increased the technical feasibility of the procedure [104]. This procedure is usually performed using a 15 mm diameter LAMS. EUS-GE is a technical complex procedure, especially on identifying a target jejunal loop and maintaining its relative position in close apposition to the stomach. Nowadays, there are three main techniques described to facilitate this limiting step during procedure: direct EUS-GE, device-assisted EUS-GE, and EUS-guided double balloon-occluded gastro-jejunostomy bypass (EPASS) [105].

A meta-analysis by Fan et al. evaluating the efficacy and safety of EUS-GE for GOO (*n* = 285) reported a pooled technical and clinical success of 92% and 90%, respectively [106]. These results were reproductible in a meta-analysis by McCarty et al. [107, 108]. Regarding safety, EUS-GE seems to have a relative low rate of AEs. Iqbal et al. [106] and McCarty et al. [108] reported a pooled incidence of AEs of 12% and 10.6%, respectively. Most reported AEs were stent misdeployment, peritonitis, bleeding, abdominal pain, and leakage. When compared to transluminal SEMS placement, EUS-GE have comparable technical and clinical effectiveness. Chandan et al. [109] reported a pooled rate for technical and clinical success of 95.2% and 93.3% in EUS-GE and 96.9% and 85.6% in SEMS. Pooled rate of reintervention was significantly lower with EUS-GE compared to SEMS (4% vs. 23.6%, *p* = 0.001); however, AEs were comparable between the two techniques. Khashab et al. [110] compared open SGJ and EUS–GE in patients with malignant GOO. Although technical success was lower with EUS-GE (86.7% vs. 100%, *p* = 0.009), there was no difference in clinical success (87% vs. 90%, *p* = 0.18). No significant statistically differences were found on recurrence and AE rates between the two groups. Kouanda et al. [111] did not found significant differences in technical or clinical success, symptom recurrence, reintervention, 30-day readmission, or 30-day mortality between EUS-GE and open SGJ. However, EUS-GE patients experienced shorter delays to resumption of oral intake and chemotherapy, had shorter lengths of stay, and reduced hospital costs. Perez-Miranda et al. [112] and Bronswijk et al. [113] compared retrospectively EUS-GE and laparoscopic SGJ, reporting no differences in technical and clinical success between groups, but EUS-GE had significantly lower rate of AEs, reduced mean time to oral intake and shorter median hospital stays.

In patients who experienced surgeries involving the stomach or the duodenum, ampulla is less readily accessible, leading to a more challenging, in some cases, unsuccessful ERCP [114]. Most cases of altered anatomy involve Roux-en-Y gastric bypass (RYGB), but also Roux-en-Y hepaticojejunostomy, choledocojejunostomy and pancreaticoduodenectomy, or Billroth II procedures. To overcome difficult ERCP in surgical altered anatomy, endoscopic ultrasound–directed transgastric ERCP (EDGE) may be used [115]. EDGE is a procedure in which the gastric pouch is connected to the excluded stomach by placing a LAMS between them (Figure 3). Then, a “traditional” ERCP can be performed by passing an ERCP endoscope through the stent in direction to duodenum to reach de ampulla [116]. The ERCP can be performed either immediately or after a delay to avoid the risk of dislodging the stent. If the patient requires an urgent or emergent ERCP, the LAMS is balloon-dilated to allow the duodenoscope to pass through, although the risk of stent dislodgement remains. To minimize this risk, some authors suggest placement of an over-the-scope clip or endoscopic suturing to anchoring the stent in place [117, 118]. Dhindsa et al. [119] evaluated EDGE, LA-ERCP, and balloon enteroscopy-assisted ERCP (BEA-ERCP) outcomes in RYGB patients. Pooled rate of technical and clinical success of EDGE was comparable to LA-ERCP but was statistically superior to BEA-ERCP. AE rates were similar between EDGE and LA-ERCP. However, when compared to BEA-ERCP, EDGE had higher incidence of AEs. LAMS migration was the most common AE (13.3%), due to immature fistula or manipulation by duodenoscope [119]. A recent study reported a persistent fistula after LAMS removal as an uncommon event, but when present its closure is recommended. Weight regain due to persistent fistula may not be a concern since most studies point towards weight loss [120]. Additionally, EDGE is more cost-effective, compared to BAE-ERCP and LA-ERCP in RYGB patients [121]. EUS-directed transgastric intervention (EDGI) is described as a novel technique for other indication rather than ERCP, permitting successful interventions in the excluded stomach and duodenum of RYGB patients [122].

Afferent loop syndrome (ALS) is an uncommon complication after Billroth II gastro-jejunostomy but may also occur after Roux-en-Y reconstruction and pancreaticoduodenectomy (Whipple procedure). ALS is defined as a mechanical obstruction leading to distension of the afferent limb secondary to the accumulation of bile, pancreatic fluid, and proximal small bowel secretions, resulting in pancreaticobiliary symptoms, deranged hepatic panel, and elevated pancreatic enzymes [123, 124]. Usually, surgery is the mainstay treatment for ALS, although it depends on the obstruction cause and patient comorbidity. In malignant causes, especially in nonsurgical candidates, endoscopic intervention for palliation may play an important role [125]. Endoscopic access to afferent loop can be obtained by endoscope or enteroscope to perform EBD or placement of double-pigtail PS/SEMS into the stricture [126]. EUS-guided transgastric access to the afferent loop has been reported in malignant ALS, where afferent loop is not completely accessible due to long enteric segment, obstructing mass, tight angulation, long stricture, or recurrence after other endoscopic techniques [127, 128]. EUS-GE can be performed using a cautery or non-cautery-enhanced LAMS. After identifying the dilated loop *via* ultrasonography, a LAMS is deployed with the distal end in the afferent loop and the proximal end in the stomach or efferent loop. Some authors recommend the use of double pigtail stents through the deployed LAMS to prevent occlusion by food or tumor ingrowth [129]. A multicenter retrospective study evaluated 18 patients who underwent EUS-GE and EUS-EE to resolve ALS secondary to malignancy. Technical success was achieved in 100%, and clinical success included resolution of symptoms (88.9%) and expedited hospital discharge (11.1%). The most common procedure was a GJ (72.2%) [130]. When compared to luminal SEMS (historical cohort), EUS-GE group had higher rates of symptom resolution and less need for reinterventions [130].

### 5.3. Benign Gastrointestinal Strictures

LAMS have recently also been considered as a viable alternative to treat benign GI strictures. The unique design of LAMS with short length, saddle shape, and wide flanges makes them less prone to migration when compared to traditional SEMS. The data on this expanded indication is still evolving. In most descriptive studies, the stricture length was <10 mm, with migration rates being comparable to FC-SEMS fixed by suture. Tan et al. performed a meta-analysis of six studies with 144 patients [131], where in the most common stricture locations were gastro-jejunal anastomosis (33.3%), esophago-gastric anastomosis (18.8%), gastro-duodenal anastomosis (17.4%), pylorus (13.2%), and colon (11.1%). The overall technical success rate was 98.3%, clinical success rate was 73.8% (Figure 4), and adverse events rate was 30.6%, with most common being stent migration (10.9%). Subgroup analysis showed higher rates of clinical success for colonic and pyloric strictures. No comparative studies of LAMS and SEMS and EBD have been reported so far.

## 6. Conclusion

The role of endoscopic stenting in the management of patients with gastrointestinal diseases has expanded greatly in recent years, both with increasing use of endoluminal and transluminal stents. BDS in the esophagus and colon show similar safety and efficacy to SEMS, with less need for reinterventions. Biliary BDS, especially helicoidal shaped, have shown favourable outcomes with minimal adverse events. DES, especially irradiating ones, might have a role in the palliative treatment of esophageal and biliary cancer by improving patients' survival. Stents also could prevent or delay the need for surgical resection and may be considered in Crohn's disease patients with colonic or ileocolonic anastomotic strictures, especially after EBD failure. Finally, LAMS have high rates of clinical success, with favourable safety profile for management of mediastinal and postsurgical abdominopelvic collections, temporary treatment of GI benign obstructions, and may also be a valid alternative for GE creation in GOO, ALS, and biliary access in RYGB patients. GI stents continue to undergo design changes to address their limitations, and further technical refinements and studies to improve and demonstrate their efficacy are needed.

## Figures and Tables

**Figure 1:** (a, b) Endoscopic images of a patient with a refractory caustic esophageal stricture who underwent placement of a 25/20/25 × 100 mm biodegradable noncovered stent. (c, d) Endoscopic images of a patient with an esophageal-jejunal anastomotic leak who underwent placement of a 28/23/28 × 100 mm biodegradable fully covered stent, covering the leak.

**Figure 2:** Patient with a mediastinal collection adjacent to the esophagus. (a) Endosonographic image showing deployment of a 10 mm diameter lumen apposing metal stent (LAMS). (b) Endoscopic image of the proximal flange placed in the esophagus. (c) Endoscopic image of the esophageal defect after LAMS removal. (d) Endoscopic image of the esophageal defect closed with endoclips.

**Figure 3:** Patient with a previous Roux-en-Y gastric bypass who presented with jaundice secondary to pancreatic cancer underwent endoscopic ultrasound directed transgastric ERCP (EDGE). (a) Fluoroscopic image showing a 20 mm diameter lumen apposing metal stent (LAMS) placed between the gastric pouch and the gastric remnant under EUS guidance. (b) Endoscopic image of the proximal flange of the LAMS in the gastric pouch.

**Figure 4:** Patient with a refractory esophago-jejunal anastomotic stricture who underwent placement of lumen apposing metal stent (LAMS) across the stricture. (a, b) Endoscopic image of the LAMS placed across the stricture. (c) Esophago-jejunal anastomotic stricture remodelling after LAMS removal.
